# CyclinD1, a prominent prognostic marker for endometrial diseases

**DOI:** 10.1186/1746-1596-8-138

**Published:** 2013-08-15

**Authors:** Shuo Liang, Kun Mu, Yan Wang, Zhiqiang Zhou, Juan Zhang, Yan Sheng, Tingguo Zhang

**Affiliations:** 1 Department of Pathology, Shandong University School of Medicine, 44#, Wenhua Xi Road, 250012 Jinan, Shandong, People's Republic of China; 2 Department of Pathology, Qilu Hospital of Shandong University, 107#, Wenhua Xi Road, 250012 Jinan, China

**Keywords:** Endometrial cancer, CyclinD1, Prognostic markers, Survival analysis

## Abstract

**Purpose:**

Alteration of CyclinD1 was suggested to relate with development of endometrial carcinogenesis before, however CyclinD1 expression is not well defined in endometrial hyperplasia lesions. We checked the relationship between its expression and clinic-pathological variables of endometrial lesions to explore the possibility for CyclinD1 as a potential diagnostic and prognostic marker.

**Methods:**

Cyclin D1 immunohistochemical analysis (IHC) was used to evaluate 201 fixed, paraffin-embedded endometrial samples which included simple hyperplasia (n = 27), atypical complex hyperplasia (ACH) (n = 41), endometrioid carcinoma (n = 103), endometrial serous carcinoma (ESC) (n = 21) and clear cell carcinoma (CCC) (n = 9). A breast cancer with known CyclinD1 expression was selected as a positive control in each immunohistochemistry run. We also performed follow-up study to estimate patients’ prognosis.

**Results:**

CyclinD1 was significantly overexpressed in atypical complex hyperplasia (ACH), endometrioid carcinoma and clear cell carcinoma (CCC). The positive signaling of CyclinD1 was showed less than 40% in simple hyperplasia and endometrial serous carcinoma (ESC). The high expression of CyclinD1 was observed in metastasis carcinoma group more significantly than non-metastasis carcinoma group. Kaplan Meier analysis demonstrated that patients with high CyclinD1 expression had an obviously poor prognosis than patients without CyclinD1 staining (*p* < 0.05). Moreover, according to multivariate Cox regression analysis, CyclinD1 expression, as crucial as metastasis, was a risk marker for overall survival rate.

**Conclusion:**

CyclinD1 exhibited a promising potential to predict the prognosis of patients with endometrial carcinoma. However, the statistical analysis demonstrated that CyclinD1 exhibited a poor ability to differentiate neoplastic lesions from non-neoplastic lesions; thus, the application of CyclinD1 only is not so credible for differentiation between benign and malignant lesions.

**Virtual slides:**

The virtual slides for this article can be found here: http://www.diagnosticpathology.diagnomx.eu/vs/1871063048950173.

## Introduction

Endometrial cancer is the most common malignancy of the female genital tract in the world and the seventh most common cause of death for women in Western Europe who suffer from cancer. Every year 7406 new cases are registered in the UK, 88 068 in the European Union and 40 102 in North America [1]. Even though the routine evaluation of estrogen receptor (ER), progesterone receptor (PR) and P53 expression in endometrial cancers are widely used, corpus uteri cancer, lacking new effective prognostic markers, still severely jeopardizes women’s health today. In that case, we are looking forward to some new diagnostic and predict indicators more accurately and credibly.

CyclinD1 (also known as BCL1) which is best known for its utility in mantle cell lymphoma diagnosis is encoded by the CCND1 gene in human beings [2-4]. As a cell -cycle regulator, CyclinD1 is essential for progression through G1 phase and is a candidate proto-oncogene [5]. Mutations, amplification and over-expression of CCND1 gene, which can alters cell cycle progression, are observed frequently in a variety of tumors and may contribute to tumorigenesis [6-9].

In this study, we investigated the expression of CyclinD1 in 5 different pathological types of endometrial diseases, including simple hyperplasia, atypical complex hyperplasia, endometrioid carcinoma, endometrial serous carcinoma and clear cell carcinoma, by immunohistochemistry. We also followed-up the patients and executed survival analysis to explore the possibility of CyclinD1as a diagnostic and prognostic marker for endometrial diseases.

## Materials and methods

### Tissue samples

Different types of endometrial samples were obtained from the Department of Pathology, Qilu Hospital affiliated to Shandong University after getting approval from an Institutional Review Board. Informed consent was obtained from all the patients. All samples were routinely fixed with 10% formaldehyde and embedded with paraffin. Histologic features of all cases were studied with hematoxylin-eosin staining (HE) and diagnosed by two clinical pathologists following established histopathologic criteria of the International Federation of Gynecology Oncology (FIGO) [10,11]. The samples include simple hyperplasia (n = 27), atypical complex hyperplasia (n = 41), endometrioid carcinoma (n = 103), serous carcinoma (n = 21) and clear cell carcinoma (n = 9). The vast majority of the carcinomas were histologically pure; where mixed, the second component constituted less than 10% of the total tumor volume.

### Immunohistochemical analysis

The streptavidin-peroxidase-biotin (SP) immunohistochemical method was performed on the paraffin sections to study the expression of CyclinD1. Briefly, 4-μm-thick paraffin-embedded tissue sections were deparaffinized with xylene and hydrated through gradient alcohols. Antigen retrieval was achieved by autoclave (170 KPa) in EDTA buffer. Followed that, the slides were treated with a blocking protein (Zhongshan Biotechnology Company, Beijing, China). The sections were incubated with mouse anti-human monoclonal CyclinD1 antibody (1:1000; Zhongshan Biotechnology Company, Beijing, China) overnight at 4°C. An avidin-biotin-peroxidase complex (Dako, Denmark) with DAB as chromogen was used for detecting antibody binding. Secondary antibody was biotinylated anti-rabbit IgG and anti-mouse IgG/IgM (Dako, Denmark) primary antibodies. Representative sections of breast carcinoma served as positive controls for CyclinD1 antibody. We replaced the CyclinD1 with non-immune IgG as negative controls.

### Evaluation of immunohistochemical staining

Cyclin D1 staining was evaluated in the glandular epithelium component in each group of simple hyperplasia, atypical complex hyperplasia, and adenocarcinoma. Two parameters were taken into consideration: the intensity of nuclear staining and the extent (percentage of positive cells). Fields for calculating percentage of immune-reactive nuclei were selected based on best tissue preservation and, where there was less artifact, wrinkling or folding. Since the immune-reactivity may not be uniform among nuclei on any given case, we determined grade as the most frequently observed pattern. The intensity of nuclear staining was graded as no staining (0), weak (1+), moderate (2+), or strong (3+). The extent was semi-quantitatively estimated with a range of 0% to 100%. Percentage was estimated by counting at least 50 nuclei and then establishing the ratio of immune-reactive nuclei to total number of nuclei multiplied by 100; percentages were rounded to the nearest 10%. When less than 10% of cells were positive, a score of 0 was used, 10% to 30% cell positivity was scored as 1, 31% to 60% positivity was scored as 2, and more than 60% positive cells was labeled as 3. However, the statistical analysis was based on the data distribution using a continuous range from 1% to 100% reactive cells.

### Survival analysis

Medical records of these 201 patients from Medical Records Center of Qilu Hospital were checked after getting the approval from Institutional Review Board. Follow-up survey was implemented by telephone calls and clinics to record the survival time of these 201 patients. We adopted Type I censoring, stopping the survey at the predetermined time September, 1st, 2012, at which point any subjects remaining are right-censored. Patients’ death from endometrial diseases were considered as the endpoint event.

### Statistical analysis

Comparison of CyclinD1 expression in different status of the endometrium was assessed by Partitioning Chi-squares and Fisher’s exact test when an expected cell value was 5 or less by PASW Statistics 18.0 software. Survival curves were created from Kaplan-Meier method with the log-rank test. Comparisons were made by Cox’s proportional hazards model regression. Results were presented in the form of hazard ratios (HR) and 95% confidence interval (95CI). A *p* < 0.05 was considered statistically significant.

## Results

### Expression of CyclinD1 in endometrial diseases

The CyclinD1 protein staining was captured specifically in endometrial glandular epithelial cell nuclei, with strong intensity of concentrated staining in endometrioid carcinoma and ESC. Nevertheless, the staining was typically of moderate in ACH and clear cell carcinoma, or weak intensity in simple hyperplasia. Representative images depicting CyclinD1 staining patterns in different lesions are illustrated in Figure 1 (A-D). The positive staining was observed in 8 of the 27 patients (30.0%) with simple hyperplasia, 49% (20/41) in atypical complex hyperplasia, 52% (54/103) in endometrioid carcinoma, 38% (8/21) in endometrial serous carcinoma and 67% (6/9) in clear cell carcinoma. A detailed summary of the data is summarized in Table 1 and illustrated in Figure 2.

**Figure 1:** **The expression of CyclinD1 tested by immunohistochemistry.** (original magnifications: 400×). **A**: CyclinD1 immunostaining in simple hyperplasia endometrial tissue, cells with a brown-stained nucleus are regarded as positive. However, negative CyclinD1 immunostaining was seen in the picture. (original magnifications: 400×); **B**:CyclinD1 staining in atypical complex hyperplasia. CyclinD1 is weakly to moderately positive in most grandular epithelium cells (original magnifications: 400×); **C**: CyclinD1 staining in endometrioid carcinoma. CyclinD1 was strongly and diffusely positive in nucleus (original magnifications: 400×). **D**: CyclinD1 staining patterns in endometrial serous carcinoma, CyclinD1 expression in ESC mostly showed a strong intensity in nucleus. (original magnifications: 400×). **E**:SET8 expression in endometrial clear cell carcinoma. The picture showed a moderate intensity of SET8 staining. (original magnifications: 400×).

**Table 1:** Expression of CyclinD1 in the tissue of endometrial lesions

**Pathological type**	**Cases assessed**	**CyclinD1**		
		**+**	**-**	Positive Rate%*
Simple hyperplasia	27	8	19	30%
Atypical complex hyperplasia	41	20	21	49%
Endometrioid carcinoma	103	54	49	52%
Endometrial serous carcinoma	21	8	13	38%
Clear cell carcinoma	9	6	3	67%

*: Grade and score by the intensity of immunoreactivity staining: 0 point for absent, 1 point for weak, 2 points for moderate and 3 points for strong; then grade by the extent of tissue staining: 0 point for no positive staining cells, 1 point for positive ratio <25%, 2 points for 25%-49%, 3 points for 50%-79% and 4 points for ≥ 80%. Finally, multiply the two score systems: ≤3 points for negative, >3 points for positive.

**Figure 2:** The comparison of the expressions of CyclinD1 in different pathological types of endometrial diseases.

### Statistical comparisons of CyclinD1 expression in endometrial lesions

Partitioning Chi-squares was applied to compare CyclinD1 expression in these five endometrial lesions individually. In order to avoid amplifying the probability to commit type I mistake, *p* value was reset as *p*’ = 1-m√ ((1)-p), ”m“ represented group numbers. In this case, *p*’ = 1-5√ ((1)-0.05) = 0.005, so we considered *p* < 0.005 as statistically significant. Although atypical complex hyperplasia, endometrioid carcinoma and clear cell carcinoma showed more positive staining compared with simple hyperplasia and endometrial serous carcinoma, the *p* value was larger than 0.005 after comparing CyclinD1 expression in five endometrial lesions with each other respectively. The expression showed no statistical significance in different endometrial lesions (p > 0.005). The corresponding statistical comparison results are listed in Table 2.

**Table 2:** Statistical comparisons of five endometrial lesions

**Parameter a vs. Parameter b**	**Positives (Parameter a)**	**Positives (Parameter b)**	**χ**^***2***^value*	*p *value*
Simple hyperplasia vs. atypical complex hyperplasia	8/27(30%)	20/41(49%)	2.465	0.116
Simple hyperplasia vs. endometrioid carcinoma	8/27(30%)	54/103(52%)	4.457	0.035
Simple hyperplasia vs. endometrial serous carcinoma	8/27(30%)	8/21(38%)	0.381	0.537
Simple hyperplasia vs. clear cell carcinoma	8/27(30%)	6/9(67%)	3.50***	0.111**
Atypical complex hyperplasia vs. endometrioid carcinoma	20/41(49%)	54/103(52%)	0.156	0.693
Atypical complex hyperplasia vs. endometrial serous carcinoma	20/41(49%)	8/21(38%)	0.640	0.424
Atypical complex hyperplasia vs. clear cell carcinoma	20/41(49%)	6/9(67%)	4.32***	0.467**
Endometrioid carcinoma vs. endometrial serous carcinoma	54/103(52%)	8/21(38%)	1.433	0.231
Endometrioid carcinoma vs. clear cell carcinoma	54/103(52%)	6/9(67%)	4.18***	0.500**
Endometrial serous carcinoma vs. clear cell carcinoma	8/21(38%)	6/9(67%)	4.20***	0.236

*: We took partitioning Chi-squares when individual comparisons were performed, in order to avoid amplifying the probability to commit type I mistake, *p* value should be reset as *p’* = 1-m√(1-p)*,* “m” represented group numbers. In this case, *p’ =* 1-5√(1-0.05) = 0.005, so we considered *p* < 0.005 as statistically significant.

**: When expected cell value was 5 or less, we used Fisher’s exact test.

***: The expected cell values were 3.50, 4.32, 4.18 and 4.20 for simple hyperplasia vs. clear cell carcinoma, atypical complex hyperplasia vs. clear cell carcinoma, endometrioid carcinoma vs. clear cell carcinoma and endometrial serous carcinoma vs. clear cell carcinoma, respectively.

### Correlation of CyclinD1 expression with the clinic-pathological features of the endometrial lesions

The clinic-pathological variables included the age, pathological type, metastasis and invasion. The ratio of positive expression of CyclinD1 was 53.0%, 50.0% and 38.0% in ≤40, 41-59, ≥60 age group respectively (p > 0.05). The positive rate of the CyclinD1 expression was 30.0%, 49.0%, 52%, 38% and 67% in simple hyperplasia, ACH, endometrioid carcinoma, ESC and CCC each (p > 0.05). The ratio of positive expression of CyclinD1 was 47.0% in the non-metastatic and 67.0% in metastatic group (*p < 0.05*), which indicated that CyclinD1 overexpression was related with tumor metastasis. The CyclinD1 expression rate was 60% in non-invasion group, 48% in <1/2 invasion group and 58% in ≥1/2 invasion group individually *(p > 0.05*), which meant that CyclinD1 overexpression had no relationship with tumor invasion. In conclusion, the expression of CyclinD1 was not correlated with age, pathological types and invasion *(p > 0.05*). However, its expression was correlated with metastasis *(p < 0.05*). The corresponding statistical results are listed in Table 3.

**Table 3:** Correlation of CyclinD1 expression with the clinicopathological variables

**Clinicopathological variables**	**Cases assessed**	**CyclinD1**				
		**+**	**-**	**Positive rate**	**χ**^***2 ***^**value**	**P value**
Age(year)						
≤40	51	27	24	0.53	2.362	0.307
41-59	103	51	52	0.50		
≥60	47	18	29	0.38		
Pathological type						
Simple hyperplasia	27	8	19	0.30	6.549	0.162
Atypical complex hyperplasia	41	20	21	0.49		
Endometrioid carcinoma	103	54	49	0.52		
Endometrial serous carcinoma	21	8	13	0.38		
Clear cell carcinoma	9	6	3	0.67		
Invasion						
None	5	3	2	0.60	1.258	0.533
<1/2	90	43	47	0.48		
≥1/2	38	22	16	0.58		
Metastasis						
No	106	50	56	0.47	4.468	0.035
Yes	27	18	9	0.67		

### Survival analysis

#### Kaplan-Meier survival curve of the expression CyclinD1 in 201 patients with endometrial diseases

Between 2007 and 2011, these 201 patients were consecutively diagnosed and treated in our hospital; median and mean ages were 52.6 and 53 years. Median follow-up period for 201 cases was 39.4 months ranging from 4 months to 68 months. The average median survival time was 42 months. The prognosis of patients were significantly determined between the two groups regarding CyclinD1 staining [log-rank(Mantel-Cox), χ^*2*^ =12.293,*p* = 0.000 ( *P*<0. 05)]. The survival curve for CyclinD1 staining group zigzagged obviously lower than CyclinD1 empty group, which is illustrated in Figure 3.

**Figure 3:** **Kaplan-Meier survival curve of the expression CyclinD1 in 201 patients with endometrial diseases.** Kaplan-Meier analysis of patients with and without CyclinD1 expression. The blue line represents the patients with CyclinD1 negative expression; the green line represents the patients with CyclinD1 positive expression. It clearly showed the patients with negative expression of CyclinD1 had higher overall survival rates than those with positive expression of CyclinD1.

#### Multivariate Cox regression analysis of CyclinD1 expression and clinic-pathological features

Multivariate Cox regression analysis demonstrated that of the factors being studies, only metastasis (HR10.198, 95% CI: 3.691–28.176, p < 0.05) and CyclinD1 staining (HR2.765, 95% CI: 1.201–6.363, p < 0.05) were significantly associated with prognosis. However, the age, pathogenic types, pathological types and invasion were not tightly associated with prognosis. The detailed information was summarized in Table 4.

**Table 4:** Multivariate cox regression analysis of CyclinD1 expression and clinicopathological variables

**Category**	**Hazard ratio**	**P-value**	**95.0%CI for HR**	
			Lower	Upper
Age	1.026	0.932	0.569	1.850
≤40				
41-59				
≥60				
Pathogenic types	1.474	0.651	0.274	7.919
I				
II				
Pathological types	1.214	0.651	0.524	2.814
Simple hyperplasia				
Atypical complex hyperplasia				
Endometrial adenocarcinoma				
Endometrial serous carcinoma				
Clear cell carcinoma				
Invasion	1.466	0.382	0.623	3.451
None				
<1/2				
≥1/2				
Metastasis	10.198	0.000	3.691	28.176
Yes				
No				
CyclinD1	2.765	0.017	1.201	6.363
+				
-				

## Discussion

Tumor is a type of general, systematic and step-by-step developing disease involving a series of factors; it is caused by the mutation of the oncogenes and disorders of some genes [12]. Endometrial carcinoma is a malignant cancer that derives from endometrial glandular epithelium. The formation of organs and tissues of female reproductive tract is through the development, evolvement and differentiation of Miller’s tube. The epithelium of Miller’s tube is characterized by a multiple differentiation potential. After birth, these undifferentiated embryonic cells retained within the germinal layer of tissue in the mature organism. So when cancers happen in the female reproductive tract organs or tissues, not only can they form the same type of cancer tissues with the original tissues, namely endometrial adenocarcinoma, [13] but also they can develop other types of cancers which derive from the multidifferentiation of Miller tubular epithelium. These types of cancers are such as endometrial serous carcinoma, clear cell carcinoma, mucinous adenocarcinoma, squamous cell carcinoma, mixed carcinoma and undifferentiated carcinoma and etc. [14,15] This situation leads to the complexity and diversity of endometrial diseases.

CCND1, as a proto-oncogene located on chromosome 11q13, has been studied in recent years. CyclinD1, the protein encoded by the gene, is originally proposed by Motokura et al, they found CyclinD1’s over expression in the parathyroid glands [16]. CyclinD1 protein plays an important and positive role during the key rate-limiting point G1 → S phase transition in the cell cycle. It can activate CDK4 or CDK6 to phosphosphorylate a series of key substrates, such as protein Rb, in that case, the transcription factors will be released to promote synthesis of DNA and accelerate the cells proliferation [17]. Thus it is an essential sensor and activator of cell cycle initiation and progression; Cyclin D1 amplification and gain copies with consequent protein over-expression have been frequently described in multiple myeloma, T cutaneous lymphomas and in solid cancer [18], such as oral squamous cell carcinoma, lung cancer, melanoma, breast cancer [19,20]. A recent study has shown that strong nuclear EGFR expression in colorectal carcinomas is associated with cyclin-D1 but not with gene EGFR amplification [21].

The results of this research showed the expression of CyclinD1 increased in the order of simple hyperplasia, ACH, endometrioid carcinoma, CCC except ESC, the statistical comparisons of these types with each other demonstrated no statistical significance (P > 0.005). However, the further analysis showed that patients with CyclinD1 expression usually accompanied by lymph node metastasis and poor prognosis (P <0. 05), this is consistent with Nikaido’s report. [21]. Thus, CyclinD1’s over expression is positively correlated with the lymph node metastasis and poor prognosis. As a positive regulator of cell cycle, CyclinD1’s over expression may lead to uncontrolled cell proliferation. Even though its expression rate increased with the level of malignancy of the endometrial lesions, it still lacks the specificity to differentiate non-neoplastic and neoplastic endometrial tissues. Therefore, we could not merely use CyclinD1 as a diagnostic marker when we confront a dilemma of distinguishing non-neoplastic and neoplastic lesions, but its application could predict the prognosis more credibly and accurately. In other words, CyclinD1 could be an applicable indicator for the prognosis of endometrial cancer. Future studies on the role of CyclinD1 of endometrial carcinogenesis are needed.

## Conclusion

In conclusion, our study demonstrated that the expression of CyclinD1 was up-regulated with the level of malignancy of the endometrial lesions; it lacks the specificity to differentiate non-neoplastic and neoplastic endometrial tissues. The results showed that the expression of CyclinD1 was tightly correlated with the metastasis of endometrial cancers. The facts above demonstrated that CyclinD1 play an important role in the formation and development of endometrial cancers. Significantly, Kaplan-Meier survival analysis and multivariate Cox regression analysis showed that CyclinD1and lymph node metastases were risk markers of overall survival; they affected the patients’ prognosis. Therefore, the evaluation of CyclinD1 may assist in predicting the prognosis of endometrial carcinoma as a supplement to ER, PR and P53. Such knowledge may help to identify new strategies for endometrial cancer treatment.

## Competing interests

The authors declare that they have no competing interests.

## Authors’ contributions

SL conceived and performed the experiments, analyzed data, and wrote the manuscript. YW did the immunohistochemical analysis. KM and TZ reviewed all the pathological slides. TZ supervised the experiments. ZZ and JZ provide technical support for slide making. SL and YS followed up the patients. All authors read and approved the final manuscript.
